The article "Variations in the Profiles of Vascular-Related Factors Among Different Sub-Types of Polycystic Ovarian Syndrome in Northern China" was published in 2021. Journal: Front Endocrinol (Lausanne).

# Variations in the Profiles of Vascular-Related Factors Among Different Sub-Types of Polycystic Ovarian Syndrome in Northern China

**DOI:** 10.3389/fendo.2020.527592

**Published:** 2021-02-26

**Authors:** Mei-mei Liu, Xiu-hui Chen, Xiu-min Lu, Fang-fang Wang, Chao Wang, Yu Liu, Pei-ling Li, Bo-tao Du, Sha Liang, Pi-dong Gong, Yu-xin Wang

**Affiliations:** Department of Gynaecology and Obstetrics, The Second Affiliated Hospital of Harbin Medical University, Harbin, China

**Keywords:** polycystic ovarian syndrome, vascular-related factors, vascular endothelial growth factor, endostatin, thrombospondin-1

## Abstract

Recently, a growing body of evidence has suggested that abnormal ovarian angiogenesis, secondary to the imbalance between various angiogenic markers, is involved in the pathogenesis of PCOS, and this has led to the use of various interventions (such as Diane-35) to restore the normal ovarian angiogenesis. Therefore, we conducted the current investigation to determine the role of such markers (endothelial growth factor (VEGF), endostatin (ES), and thrombospondin-1 (TSP-1)) in the pathogenesis of PCOS along with the associated changes in ovarian blood flow in patients with PCOS compared to healthy controls, both before and after a course of oral contraception. A total of 381 patients with PCOS and 98 healthy females of childbearing age were recruited from July 2014 to June 2017 at the Reproductive Center of the Second Affiliated Hospital of Harbin Medical University. The serum levels of VEGF, ES, and TSP-1 were determined by enzyme-linked immunosorbent assay, while ovarian perfusion was measured by the pulsatility index (PI) and resistance index (RI) by using transvaginal color Doppler ultrasound. Repeated analyses were carried out after 3 months of Diane-35 treatment. Post-treatment serum levels of luteinizing hormone (LH)/follicle stimulating hormone (FSH) ratio of patients with PCOS decreased significantly (P <0.05). The RI values of most PCOS patients increased after treatment (P<0.05), while PI was significantly increased in all patients (P<0.05). However, variable changes in the serum levels of TSP-1, VEGF, and ES after treatment were observed. Serum VEGF levels showed a negative correlation with serum LH/FSH ratio, T concentration, and ES (P <0.05), while ES levels were negatively correlated with serum T concentrations only (P<0.05). The markers of angiogenesis (VEGF, ES, and TSP-1) were expressed differently among PCOS patients, who also responded differently to the same course of Diane-35 treatment. This field still warrants further investigation to reach a more definitive conclusion.

## Introduction

Polycystic ovary syndrome (PCOS), a gynecological and endocrinal disorder in women, has been recently characterized by the disruption of ovarian blood flow and angiogenesis (1). The prevalence of PCOS is 5%–7% among women of childbearing age (19–25 years). Despite being variable in different populations, the main presentations of PCOS include ovulation disorders (oligo or amenorrhea), hyperandrogenism (HA), insulin resistance (IR), and metabolic or psychological disturbances (2, 3). To date, the pathogenesis of PCOS has not been well-studied. However, it has been proposed that ovarian angiogenesis plays a crucial role in the pathogenesis of PCOS, given the fact that the formation and regression of blood vessels are mandatory for proper follicle maturation, ovulation, and corpus luteum formation (1). Therefore, it was proposed that such vascular alterations, controlled by various angiogenic markers, would be responsible for the ovarian features of PCOS (4).

Vascular endothelial growth factor (VEGF), which is responsible for promoting the proliferation of vascular endothelial cells and regulating vascular permeability, is of great importance in follicular development (5). Endostatin (ES), an anti-angiogenic factor, interferes with the pro-angiogenic action of VEGF and inhibits the proliferation of endothelial cells (ECs) while suppressing the formation of new blood vessels (6). Thrombin sensitive protein-1 (TSP-1), known as thrombospondin-1, is also an important inhibitor of angiogenesis, acting by inducing apoptosis in ECs by targeting VEGF (6).

A growing body of evidence suggests that VEGF, ES, and TSP-1 are abnormally expressed in patients with PCOS (7, 8).

Moreover, it is proposed that the disruption of normal ovarian angiogenesis, secondary to the imbalance between angiogenic and anti-angiogenic factors, is responsible for the occurrence of several pathologies in PCOS, including abnormal follicle development, increased quantity of small follicles, anovulation, and cyst formation (1). Consequently, various interventions (such as oral contraceptive pills and metformin) have been proposed as therapeutic options for PCOS, acting by restoring the normal ovarian angiogenesis (9, 10).

Therefore, we conducted this study to determine the role of alterations in the expression of the aforementioned angiogenic markers in the pathogenesis of PCOS, along with the associated changes in ovarian blood flow. We also investigated the changes in the expression of these markers following the use of Diane-35 in women with PCOS.

## Materials and Methods

### Subjects

In this prospective case-control study recruited 381 patients with PCOS who attended the Reproductive Center of the Second Affiliated Hospital of Harbin Medical University from July 2014 to June 2017. In addition, we included 98 healthy women of childbearing age, who received intracytoplasmic sperm injection due to male factor infertility as the control group. This research is approved by the Ethics Committee of the Second Affiliated Hospital of Harbin Medical University (KY2018-043).

### Inclusion Criteria

We followed the recommendations of the Rotterdam International Conference (11) and the Chinese PCOS diagnostic criteria (2011) (12) in diagnosing women with PCOS. The diagnosis of PCOS was reached if 2 or 3 items of the following criteria were fulfilled:

(1) Clinical manifestations of oligo and/or anovulation, which included:
a. Oligomenorrhea: the menstrual cycle is from 35 days to 6 months per year.
b. Amenorrhea: either secondary amenorrhea (menopause period ≥ 6 months) or primary amenorrhea (no menarche at 16 years old).
c. Irregular uterine bleeding: irregular menstrual cycle or period or menstrual flow.
(2) Clinical and/or biochemical signs of hyperandrogenism, which included:
a. Symptoms of HA: acne, hypersexual hair, obesity, black acanthosis, etc.
b. Biochemical determination of serum reproductive hormone concentration: biochemical HA
The laboratory diagnosis of HA in our center was determined if the total serum testosterone level was > 0.48 ng/ml.
(3) Ultrasound examination showing polycystic ovarian changes:
a. ≥12 follicles with a diameter of 2-9 mm in one or both ovaries, and/or:
b. ovarian volume ≥10 cm3 [ovary volume is 0.5 × longitudinal diameter (cm) × transverse diameter (cm) × forward and backward diameter (cm)].

Patients were included when they fulfilled at least two of the mentioned criteria, with the exclusion of other causes at the same time. Moreover, patients with other causes of hyperandrogenism were also excluded, such as abnormal thyroid function, hyperprolactinemia, delayed-type adrenal hyperplasia, 21-hydroxylase deficiency, Cushing syndrome, schizophrenia syndrome, primary hypoovarian dysfunction, or premature ovarian failure, ovarian or adrenal androgen-producing tumors, and functional hypothalamic amenorrhea.

Patients were then stratified according to the presenting manifestations into four groups of PCOS phenotypes: group A (patients who fulfilled criteria 1, 2, and 3), group B (patients who fulfilled criteria 1 and 3), group C (patients who fulfilled criteria 1 and 2), and group D (patients who fulfilled criteria 2 and 3).

On the other hand, the inclusion criteria of the normal control group were as follows: (1) healthy women of childbearing age, who are unable to bear children due to male factor infertility, (2) women with normal menstruation and without any clinical manifestations of PCOS, (3) women with no endocrinal disorders, such as abnormal sex hormone levels, abnormal oral glucose tolerance test (OGTT), or insulin resistance (IR), and (4) women with no evidence of abnormal changes in the uterus or the ovaries based on ultrasound examination.

### Exclusion Criteria

Individuals in the control group were excluded if they had systemic inflammatory diseases, thyroid disease, hyperprolactinemia, adrenal disease, hypertension, diabetes, or other complications. Those who had used hormonal drugs in the past 6 months prior to participation in the study were also excluded.

### Collection of Blood Samples

All study participants were enrolled at the early follicular stage (days 2–4 of the menstrual cycle). If no dominant follicles were found in both ovaries by transvaginal ultrasound examination, a 5 ml sample of peripheral venous blood was collected from fasting patients in the morning and placed in a polypropylene microcentrifuge tube. The tube contents were centrifuged at 2,000 r/min, and the serum was then frozen and stored in a refrigerator at -20°C for later use.

### Determination of Sex Hormone Levels

Peripheral venipuncture, during the early follicular phase of the menstrual cycle (days 2-4), was done to collect blood samples for hormonal level estimation following overnight fasting. Electrochemiluminescence immunoassay was used to measure the levels of sex hormones, including luteinizing hormone (LH), follicle-stimulating hormone (FSH), and total testosterone (T). The corresponding sex hormone kits were purchased from Tosoh Corporation, Japan. The remaining serum was stored in a refrigerator at -20°C for later use.

### Determination of Serum VEGF, ES, and TSP-1 Levels

The primary outcome of our study was to determine the changes in the expression of angiogenic markers (VEGF, ES, and TSP-1) along with the associated alterations in ovarian blood flow) in women with PCOS compared to healthy controls before and after a course of Diane-35 treatment.

The serum levels of VEGF, ES, and TSP-1 were measured from the remaining patients’ serum by immunosorbent assay (ELISA) following the manufacturer’s manual (AIA-2000 automatic immunoluminescence analyzer Japan Tosoh Co. Ltd). ELISA kits were purchased from (Shanghai Baili Biotechnology Co. Ltd.) and (Nanjing Heikeer Biotechnology Co. Ltd, Japan).

### Measurement of Ovarian Interstitial Blood Flow

On the day of blood collection, transvaginal color Doppler ultrasound was used to monitor ovarian interstitial blood flow (ProSound α7 Doppler color ultrasound Aloca, Japan). Pulsatility (PI) and resistance indices (RI) were used to measure ovarian blood flow. This process was conducted by the same clinician. In each case, the volume of ovarian interstitial blood flow on each side was taken three times, and the average value was then calculated and analyzed.

### Compound Cyproterone (Diane-35) Treatment

Patients with PCOS received oral Diane-35 on the 5th day of their menstrual periods. Diane-35 is made up of Ethinylestradiol (35 μg) and Cyproterone acetate (2 mg), and patients were given this drug at a dose of one tablet a day for 21 days per cycle. They continued receiving this medication for three successive cycles. After that, the serum levels of the aforementioned markers were reassessed.

### Statistical Analysis

We used the Statistical Package for Social Sciences (SPSS) software (Version 23.0) to conduct our analyses. Data were expressed as means ± standard deviations $\left(\bar{\chi }\pm \text{SD}\right)$. Normality (Shapiro-Wilk) and homogeneity (Levene) tests were conducted to test the distribution of the data. If the data were normally and homogeneously distributed, the differences among multiple groups were analyzed through a one-way analysis of variance (ANOVA). Post-hoc comparisons of each group were performed using the LSD test, while the Paired t-test was used to draw comparisons between groups before and after treatment. The two-tailed Pearson test was used to establish correlations between analyzed variables. A value of P <0.05 was considered the cut-off value for statistical significance.

## Results

### Demographic and Clinical Characteristics

A total of 381 patients with PCOS were included in the case group, with 94, 103, 95, and 89 patients in groups A, B, C, and D, respectively. The mean age in each group did not differ significantly from the control group (P=0.337). However, baseline BMI was significantly higher in all PCOS groups compared to control (P <0.05). Serum LH/FSH ratio and T levels in all groups of PCOS patients were significantly higher than those in the control group (P <0.05). Ovarian artery PI and RI values were significantly lower in patients with PCOS in all groups compared to the control group (P <0.05). Similarly, serum TSP-1 levels in all PCOS groups were significantly lower than the control group (P <0.05). On the other hand, serum ES levels in all PCOS groups were significantly higher than those recorded in the control group (P <0.05). Noteworthy, serum VEGF levels were significantly higher in group B only when compared to the control group (980.5 vs. 620.4, P <0.001). On the other hand, serum VEGF levels in groups A, C, and D were lower compared to the control group; however, this difference did not reach statistical significance (P >0.05) (**Table 1**). **Figure 1** shows the ultrasonic images of ovarian blood flow and the reported PI value during the assessment before Diane-35 treatment in the control group and the various PCOS phenotypes (A, B, and D).

**Table 1:** Demographic characteristics and laboratory parameters of included patients in each group at baseline.

Variable	PCOS groups				Control (N=98)	P-value
	Group A (N=94)	Group B (N=103)	Group C (N=95)	Group D (N=89)		
**Age (years)**	25.4 ± 3.5	24.7 ± 3.2	25.1 ± 3.2	24.6 ± 3.0	25.4 ± 3.9	0.337
**BMI (Kg/m2)**	26.2 ± 4.1*	25.2 ± 4.7*	25.2 ± 4.3*	25.2 ± 4.5*	22.1 ± 3.8	0.000
**LH/FSH ratio**	2.5 ± 1.0*	2.0 ± 0.9*^#^	2.9 ± 1.3*^#&^	2.8 ± 1.4*^&^	1.5 ± 1.0	0.000
**T (ng/ml)**	0.6 ± 0.2*	0.3 ± 0.1^#^	0.5 ± 0.1*^#&^	0.5 ± 0.1*^#&^	0.3 ± 0.1	0.000
**RI**	0.6 ± 0.2*	0.5 ± 0.2*	0.6 ± 0.2*^&^	0.5 ± 0.2*^$^	0.7 ± 0.2	0.000
**PI**	1.7 ± 0.8*	1.4 ± 0.4*^#^	1.5 ± 0.4*^#^	1.5 ± 0.4*^#^	2.1 ± 0.8	0.000
**TSP-1 (ng/ml)**	161.0 ± 24.5*	166.4 ± 24.6*	179.3 ± 23.6*^#&^	169.5 ± 15.8*^#$^	189.4 ± 23.1	0.000
**VEGF (pg/ml)**	606.5 ± 132.3	980.5 ± 174.6*^#^	595.8 ± 118.2&	581.2 ± 139.0^&^	620.4 ± 108.1	0.000
**ES (ng/ml)**	269.8 ± 25.6*	289.2 ± 26.8*^#^	256.1 ± 23.1*^#^&	273.0 ± 34.0*^&$^	177.8 ± 21.9	0.000
**HOMA-IR**	5.3 ± 3.1*	4.9 ± 2.0*	5.3 ± 2.2*	3.8 ± 1.4*^#&$^	2.2 ± 0.6	0.000

*significant difference compared to control; ^#^significant difference compared to group A; ^&^significant difference compared to group B; ^$^significant difference compared to group D; BMI, Body Mass Index; LH, Luteinizing Hormone; FSH, Follicle Stimulating Hormone; RI, Resistance Index; PI, Pulsatility Index; TSP-1, Thrombospondin-1; VEGF, Vascular Endothelial Growth Factor; ES, Endostatin; HOMA-IR, Homeostasis Model Assessment of Insulin Resistance.

**Figure 1:** Ultrasound recording of the ovarian blood flow in: **(A)** a normal female; **(B–D)** in patients with PCOS stratified into phenotypes A, B, and D, respectively, as described in the methods section.

### Clinical and Biochemical Characteristics After Diane-35 Treatment

Following the treatment with Diane-35, the serum levels of LH/FSH ratio in all PCOS groups were significantly reduced compared to pre-treatment levels (P <0.05). Similarly, serum T concentration was significantly lower after treatment in all groups except for group B, which did not show statistical significance. After treatment, both PI and RI values were significantly increased in all PCOS groups compared to pre-treatment levels; however, group C did not show any statistically significant difference regarding RI. In the same context, serum TSP-1 indices were significantly increased in groups A, B, and D after treatment (P<0.05). In contrast, serum VEGF levels were significantly reduced after treatment in groups B and C only (P< 0.05). Moreover, serum ES levels in groups A, B, and C were significantly decreased after treatment (P <0.05) (**Table 2**). **Figure 2** shows the ultrasonic images of ovarian blood flow and the reported PI value after a course of Diane-35 treatment in the various PCOS phenotypes (A-D).

**Table 2:** Changes in ovarian functions among PCOS patients following a course of Diane-35 treatment.

Parameter	Group A (N = 94)			Group B (N = 103)			Group C (N = 95)			Group D (N = 89)		
	Before treatment	After treatment	P	Before treatment	After treatment	P	Before treatment	After treatment	P	Before treatment	After treatment	P
**LH/FSH ratio**	2.51 ± 0.96	2.04 ± 0.61	0.000	2.03 ± 0.91	1.61 ± 0.43	0.000	2.87 ± 1.30	1.70 ± 0.5	0.000	2.75 ± 1.43	1.76 ± 0.52	0.000
**T (ng/ml)**	0.59 ± 0.17	0.45 ± 0.08	0.000	0.28 ± 0.09	0.29 ± 0.08	0.479	0.51 ± 0.09	0.39 ± 0.10	0.000	0.50 ± 0.09	0.40 ± 0.4	0.000
**RI**	0.57 ± 0.24	0.87 ± 0.22	0.000	0.52 ± 0.17	0.73 ± 0.22	0.000	0.59 ± 0.17	0.61 ± 0.20	0.544	0.53 ± 0.19	0.72 ± 0.22	0.000
**PI**	1.72 ± 0.76	1.93 ± 0.28	0.012	1.36 ± 0.41	1.91 ± 0.42	0.000	1.48 ± 0.43	1.88 ± 0.61	0.000	1.51 ± 0.39	1.90 ± 0.50	0.000
**TSP-1 (ng/ml)**	161.0 ± 24.5	180.62 ± 20.93	0.000	166.4 ± 24.6	174.13 ± 20.45	0.022	179.27 ± 23.55	182.56 ± 22.79	0.297	169.49 ± 15.83	175.72 ± 21.91	0.021
**VEGF (pg/ml)**	606.5 ± 132.3	589.48 ± 123.47	0.368	980.5 ± 174.6	896.34 ± 120.72	0.000	595.79 ± 118.20	553.95 ± 132.05	0.038	581.17 ± 139.02	550.79 ± 100.54	0.074
**ES (ng/ml)**	269.8 ± 25.6	258.25 ± 25.37	0.003	289.2 ± 26.8	229.52 ± 25.70	0.000	256.07 ± 23.09	217.85 ± 24.67	0.000	273.98 ± 34.03	265.69 ± 27.82	0.136

BMI, body mass index; LH, luteinizing hormone; FSH, follicle stimulating hormone; RI, Resistance Index; PI, Pulsatility Index; TSP-1, thrombospondin-1; VEGF, vascular endothelial growth factor; ES, endostatin.

**Figure 2:** Images of ultrasound recordings of ovarian blood flow among PCOS patients after Diane-35 treatment. Images **(A–D)** are of representative patients in groups **(A–D)**, as described in the methods section.

### Correlations Between Biological Indicators and Ovarian Blood Flow

Serum VEGF levels were found to be negatively correlated with serum LH/FSH ratio (r= -0.180), T concentrations (r= -0.581), and PI (r= -0.138) (P <0.05). However, we found that VEGF levels were positively correlated with ES levels (r= 0.266, P <0.05). On the other hand, ES levels were only negatively correlated with serum T concentrations (r= -0.237, P <0.05). There were no correlations between serum TSP-1 levels with any other biological indicators, PI, or RI (P >0.05). None of the three biomarkers depicted a correlation with RI (**Figure 3**).

**Figure 3:** Scatter plots for the correlation analysis of the expression of serum VEGF, ES and serum sex hormones among PCOS patients**. (A)** Correlation analysis between serum VEGF levels and serum T concentrations (r = -0.581, P <0.001); **(B)** Correlation analysis between serum VEGF levels and PI (r = -0.138, P =0.007); **(C)** Correlation analysis between serum ES levels and serum T concentrations (r = -0.237, P <0.001); **(D)** Correlation analysis between serum VEGF levels and LH/FSH ratio (r = -0.180, P <0.001); **(E)** Correlation analysis between serum ES levels and serum VEGF levels (r = 0.266, P <0.001). T, Testosterone; VEGF, Vascular Endothelial Growth Factor; ES, Endostatin; LH/FSH, Luteinizing Hormone/Follicular Stimulating Hormone; PI, Pulsatility Index; P, P-value.

## Discussion

Ovarian blood flow perfusion reflects the phases of follicular development and the accompanying hormonal changes. This can be monitored by the occurrence of ovulation as well as the formation and degradation of the corpus luteum (13). The hemodynamic parameters RI and PI reflect the resistance of ovarian arterial blood flow, where lower values suggest a greater degree of perfusion (14). In this study, we found that the ovarian interstitial blood flow in patients with PCOS was significantly increased (lower RI and PI values) compared to healthy controls. Going in line with other studies, the ultrasound results from our study revealed that ovarian interstitial blood flow, which was rich and with round and blunt peaks, was also characterized with high speed and low-resistance (8, 15, 16).

It has been reported that changes in ovarian blood flow are associated with high serum LH and insulin levels in patients with PCOS (17). Additionally, it is speculated that the abnormal perfusion of ovarian blood flow observed among PCOS patients is closely related to endocrinal disorders, which may be implicated in the ovulation disorders displayed by patients with PCOS (18). Moreover, abnormalities in ovarian angiogenesis that were observed in many patients with PCOS are accompanied by changes in the expression of various cytokines, which are known to regulate angiogenesis (7).

For instance, VEGF is a highly effective angiogenic factor, promoting the proliferation of vascular endothelial cells and tube formation through the action of tyrosine kinase receptors (19). VEGF plays a role in maintaining the dynamic balance of blood flow around the follicles (19). It increases the capillary permeability with subsequent extravasation of plasma proteins, which results in the increase of the ovarian matrix. This, in turn, influences the development and maturation of follicles (20). It also acts by promoting endothelial proliferation, migration, and survival (21). Some studies reported that increased ovarian vascularity is associated with an increase in serum VEGF levels in patients with PCOS (22, 23). In our study, VEGF levels of PCOS subtypes were variable compared to the control group. All PCOS subtypes, except for subtype B, had lower mean VEGF values compared to the control group; however, these differences did not reach statistical significance, which may be attributable to the small sample size of each group. This goes in line with the literature (24). Of note, PCOS subtype B (normal androgen levels) had significantly higher mean VEGF levels compared to the control group as well as other PCOS subtypes. This is inconsistent with the current evidence that suggests that increased androgens activate hypoxia-inducible factor 1 (HIF1) (25, 26), a documented transcriptional activator of VEGF (27), and this androgen receptor-mediated effect is amplified in hypoxic conditions (28, 29). Various factors have been proposed to affect VEGF levels in women with PCOS. For example, vitamin D supplementation reduces VEGF levels in women with PCOS (24). This potential confounder was not studied in our study, and the heterogeneity between our findings and the available evidence should be thoroughly investigated in future research.

ES, on the other hand, is a potent inhibitor of angiogenesis. The biological actions of ES include inhibition of angiogenesis of tumor cells and induction of apoptosis. As a result, ES inhibits the formation of new blood vessels; however, it has no effect on present healthy vessels (30). Studies have suggested that ES can specifically inhibit the proliferation of vascular endothelial cells and block the pro-angiogenic effect of VEGF (31). Moreover, ES can also inhibit endothelial cell nitric oxide synthase (eNOS) phosphorylation, induce eNOS inactivation, and reduce VEGF-induced NO synthesis. These effects lead to the inhibition of VEGF-mediated angiogenesis and vascular permeability (32). VEGF acts mainly by binding to endothelial cell receptors, mainly VEGFR-1 (vascular endothelial growth factor receptor 1), which is also known as soluble fms-like tyrosine kinase-1 (sFlt-1). On the other hand, ES inhibits angiogenesis by directly binding to sFlt-1 and interfering with VEGF-sFlt-1 interaction (33). The present study found a positive correlation between serum ES and VEGF levels among patients with PCOS, indicating that the two molecules have an important synergistic relationship in regulating angiogenesis. Since abnormally elevated VEGF promotes angiogenesis, homeostatic regulation will prompt the production of ES (angiogenesis inhibitor) to counteract the accelerated event of angiogenesis. This would explain the significant increase in ES in PCOS patients (8). However, this compensatory effect does not restore the internal environment of the body to a normal physiological state (8). The dysregulation propagates abnormal vascularization and increased perfusion of the ovarian stroma (4).

The anti-angiogenic glycoprotein molecule TSP-1 is found in the extracellular matrix of both normal and tumor cells (34). The biological actions of TSP-1 arise from binding to its receptors and promoting apoptosis as well as cellular migration. TSP-1 has been reported to indirectly affect the biological activity of VEGF (34). The anti-angiogenic effects of TSP-1 have been confirmed in patients with endometriosis (35). Patients with chocolate cysts have been demonstrated to have high levels of TSP-1 and low levels of VEGF in their ovarian tissues (36). An imbalance in the expression of TSP-1 and VEGF may be a potential cause of endometriosis (35). Lower serum TSP-1 levels have been reported in PCOS patients compared to the normal population.

On the other hand, PCOS patients having insulin resistance have displayed a higher TSP-1 level compared to patients with insulin resistance who do not have PCOS (36, 37). Additionally, TSP-1 is known to be expressed in normal ovarian tissues, while TSP-1, together with its receptor CD36, plays an important regulatory role in ovarian function, including follicular growth, luteal formation, and ovarian angiogenesis (38). Based on the documented biological activities of TSP-1, it is thus speculated that the molecule plays an important role in the development of PCOS. The vascular phenomena observed in patients with PCOS may, therefore, be contributed to both TSP-1 and VEGF expression.

In our study, we noted that the LH/FSH ratio was significantly higher in all PCOS subtypes compared to healthy controls. This would help in the identification of PCOS patients from normal women. A recent case-control study (441 PCOS women and 422 non-PCOS women) was conducted to examine the diagnostic ability of the LH/FSH ratio in the identification of PCOS cases (39). An optimum LH/FSH ratio cut-off value of 1.33 was significant to diagnose PCOS (area under curve = 0.867). Furthermore, a one-unit increase in LH/FSH ratio is associated with an increase in the risk of PCOS by 14.43 folds (95% CI= 9.30–22.39). Despite the fact that this biomarker alone is not sufficient for a proper diagnosis of PCOS, the combination of various endocrine factors (such as LH and LH/FSH ratio) along with BMI, other anthropometric measures, and clinical features may provide an extra value in the establishment of a PCOS diagnosis.

The resolution of dysregulated angiogenesis, in general, as a potential therapeutic option has witnessed increasingly rapid advances in many pathological diseases, such as cancer (40, 41), inflammatory conditions, retinal diseases, and age-related macular degeneration (42–44). Since dysregulated ovarian angiogenesis is a main feature of PCOS, restoring normal angiogenesis has been suggested as a possible therapeutic approach for PCOS to improve ovulation and fertility in affected populations. In this context, a growing body of evidence has investigated the effect of various therapeutic approaches on ovarian angiogenesis, including laparoscopic ovarian drilling (45), metformin (10), VEGF inhibitor (46), platelet-derived growth factor BB (PDGFBB) (47), and oral contraceptive pills (9). In a recent case-control study, it was observed that both RI and PI were significantly increased in healthy women (control group), as well as in women who received oral contraceptive pills (30 mcg Ethinyl estradiol and drospirenone 3 mg for 3 months) (9). This goes in line with our observation. In our study, all PCOS subtypes had significantly lower PI and RI at baseline (before treatment) compared to the control group. After a 3-month course of Diane-35 (Ethinyl estradiol), we noted that both PI and RI values increased in all groups compared to pre-treatment levels. These observations of low levels of Doppler measurements may reflect increased ovarian stromal vascularization in PCOS patients (45, 48–52). A few reports have studied the effects of OCP on ovarian blood flow in women with PCOS, and they have reported that OCP is correlated with reduced ovarian vasculature (49, 53). The reduction in PI and RI values at baseline in patients with PCOS could be explained by the main pathophysiologic mechanism of PCOS, as discussed above, with the involvement of various angiogenic markers in this process. Moreover, it has been proposed that higher levels of IR are of great importance in the regulation of ovarian vascularity in women with PCOS *via* the increase in androgen production and angiogenesis (48, 50, 52). Another explanation for the reduced ovarian angiogenesis (increased PI and RI) could be the associated increase in the expression of the anti-angiogenic factor TSP-1, which increased significantly after Diane-35 treatment, despite the lack of a significant correlation between both markers in our analysis, probably due to the small sample size. These observations suggest that the use of Diane-35 treatment could be a potential therapeutic option for restoring normal angiogenesis in patients with PCOS.

Our study provides a helpful insight into the pathogenesis of PCOS by the variable expression of pro-angiogenic and anti-angiogenic factors. We noted the ovarian blood flow indices (PI and RI), as well as TSP-1 levels, were reduced in PCOS patients compared to controls. On the other hand, ES levels were increased in all PCOS patients, while VEGF was only significantly increased in a subset of PCOS patients with hyperandrogenemia, as compared with healthy controls. That being said, our study had several limitations, the most important of which is the small number of included participants in each group, which was not sufficient enough to detect statically significant differences. Also, all lab values were monitored by a single clinician who was not blinded to the status of the patient. An important point to consider is that our results could be confounded by many un-analyzed variables, and therefore, more studies of larger sample sizes are still warranted to reach a definitive conclusion. Based on the aforementioned limitations, our findings should be interpreted with caution.

In conclusion, our study demonstrates that the dysregulation of ovarian angiogenesis is a central feature in the pathogenesis of PCOS, contributing to various phenotypes of the disease. Compared to healthy controls, low levels of Doppler measurements and changes in the expression level of various angiogenic and anti-angiogenic markers are also seen in women with PCOS. Diane-35 therapy resulted in an increase in Doppler measurements and TSP-1 biomarker levels in most PCOS phenotypes. However, variable observations regarding the expression levels of VEGF and ES were noted following a course of Diane-35 treatment. Finally, the imbalance of these biomarkers plays a role in the pathogenesis of PCOS, and the use of therapeutic options that affect ovarian angiogenesis would be of great importance in restoring normal follicular development, ovulation, and corpus luteum formation. More studies are still warranted to clarify the role of angiogenesis in different PCOS phenotypes and to develop new potential therapeutic strategies.

## Data Availability Statement

The original contributions presented in the study are included in the article/supplementary material. Further inquiries can be directed to the corresponding author.

## Ethics Statement

The studies involving human participants were reviewed and approved by Second Affiliated Hospital of Harbin Medical University. The patients/participants provided their written informed consent to participate in this study.

## Author Contributions

M-ML wrote and approved the manuscript. X-HC revised the manuscript. X-ML, F-FW, CW, YL, and SL collected data. P-LL, B-TD, Y-XW, and P-DG analyzed the patient data. All authors contributed to the article and approved the submitted version.

## Funding

This study was supported by the Joint Guiding Project of Natural Science Foundation of Heilongjiang Province (no. LH2019H070) and the Research Fund for Young and Middle-Aged Innovative Science, the Second Affiliated Hospital of Harbin Medical University (no. KYCX 2018-03).

## Conflict of Interest

The authors declare that the research was conducted in the absence of any commercial or financial relationships that could be construed as a potential conflict of interest.
